The article "Comparison of Effectiveness as well as Advantages and Disadvantages of Different Dimensions of Hysterosalpingo-Contrast Sonography for Diagnosis of Lesions Associated with Female Infertility" was retracted in 2023. Reasons: signs of a paper mill; compromised peer review; unreliable results or conclusions.

# Comparison of Effectiveness as well as Advantages and Disadvantages of Different Dimensions of Hysterosalpingo-Contrast Sonography for Diagnosis of Lesions Associated with Female Infertility

**DOI:** 10.1155/2022/7508880

**Published:** 2022-09-17

**Authors:** Rudi Pei

**Affiliations:** Department of Ultrasound, Pukou Branch Hospital of Jiangsu People's Hospital, Nanjing Pukou Central Hospital, Nanjing, Jiangsu 211800, China

## Abstract

**Methods:**

Forty subjects who underwent routine two-dimensional (2D) vaginal ultrasound, three-dimensional HyCoSy (3D-HyCoSy), and four-dimensional HyCoSy (4D-HyCoSy) examinations from January 2021 to July 2022 at the ultrasound department of Pukou Branch of Jiangsu Province Hospital were enrolled to this study. Fallopian tubal recanalization by hydrotubation (FTRH) was used as the gold standard to compare the efficacy of 2D vaginal ultrasound, 3D-HyCoSy, and 4D-HyCoSy in assessing the subjects for the presence of polyps, myomas, and other occupants in the uterine cavity or uterine adhesions.

**Results:**

A total of 18 cases of uterine cavity lesions, 11 of pelvic lesions, and 11 of ovarian lesions were identified by FTRH, while 80 fallopian tubes were found in 40 patients and 71 tubal obstructions were detected by FTRH. Vaginal ultrasound assessment of uterine cavity, pelvis, ovarian lesions, and tubal obstruction was moderately consistent with FTRH (Kappa = 0.616, 0.673, 0.654, and 0.640), 3D-HyCoSy was in good agreement with FTRH (Kappa = 0.812, 0.910, 0.906, and 0.894), and 4D-HyCoSy was in good agreement with FTRH (Kappa = 0.914, 0.903, 1.000, and 0.942), with 4D-HyCoSy being in good agreement with FTRH had the highest agreement.

**Conclusion:**

4D-HyCoSy can be used as an effective tool for clinical diagnosis of female tubal obstruction infertility and provide a reference basis for the design of subsequent clinical treatment plans.

## 1. Introduction

With social pressures and changes in lifestyle habits, the incidence of female infertility has increased in recent years [1]. Surveys show that more than 300,000 new cases of infertility have been reported worldwide in 2020, an increase of 4-5 times compared to 2000 [2]. The occurrence of infertility not only increases a woman's mental stress, but also brings great economic pressure, which seriously affects the normal life of patients [3]. Currently, the clinical causes of infertility are extremely complex and can be caused by lesions of the uterus, fallopian tubes, and ovaries, among which tubal factors are the most common, accounting for about 25-50% of all patients [4]. Infertile women often have symptoms such as obesity, chronic lower abdominal pain, and obvious dysmenorrhea, and many infertile women do not have any clinical symptoms [5]. There is no way to diagnose the cause of infertility based on these clinical symptoms alone. A series of tests are needed to help diagnosis. Therefore, how to make timely and accurate assessment of the patency of the fallopian tubes in infertile women is of great importance in the clinical management of infertility [6]. Currently, there are various clinical methods for the evaluation of tubal obstruction, such as hysterosalpingography under X-ray, uterine tubal fluid, FTRH, and hysterosalpingography under ultrasound [7]. Among them, fallopian tubal recanalization by hydrotubation (FTRH) is used as the most effective and accurate way to diagnose tubal patency and is the gold standard for infertility testing [8]. However, FTRH is extremely invasive and the test is expensive and carries a greater risk of use, which limits it from being the first choice for infertility testing [9]. Because of this, the search for an effective, safe, and accurate test is a hot topic in modern infertility diagnosis and treatment.

Hysterosalpingo-contrast sonography (HyCoSy) is a noninvasive, radiation-free test that did not gain clinical attention in the early stages of development because of unsatisfactory visualization and radiation exposure [10]. With the continuous development of contrast agents and ultrasonography technology, three-dimensional HyCoSy (3D-HyCoSy) and four-dimensional HyCoSy (4D-HyCoSy) have been developed, and the quality of their image quality has been improved dramatically on the basis of the original HyCoSy, which has been preliminarily confirmed for morphological assessment of the fallopian tubes. For example, Hong's research shows that 3D-HyCoSy can accurately assess the state of pelvic adhesions in women and can be used for the assessment of tubal obstruction in women with infertility [11]. Pan said that 4D-HyCoSy has a very comprehensive imaging effect on women's fallopian tubes, pelvis, and uterus. Endometrial thickness, fallopian tube wall, ovarian motility, etc. can be clearly observed, which has important research significance for evaluating female infertility [12]. Since HyCoSy is noninvasive, has no allergy and anesthesia risks, is radiation-free, and allows conception within a short period of time after the test, if its role in infertility evaluation can be confirmed, it will be an important enhancement for the future treatment of infertility.

Therefore, this study aims to provide a reference for the future clinical application of HyCoSy by comparing the advantages and disadvantages of different dimensions of HyCoSy for the diagnosis of female infertility.

## 2. Materials and Methods

### 2.1. Study Area

The study was carried out at the Department of Ultrasound, Pukou Branch Hospital of Jiangsu People's Hospital, from January 2021 to July 2022.

### 2.2. Research Subjects

Forty subjects who underwent routine two-dimensional (2D) vaginal ultrasound, 3D-HyCoSy, and 4D-HyCoSy examinations in the Ultrasound Department of Pukou Branch of Jiangsu Province Hospital from January 2021 to July 2022 were enrolled to retrospective analysis, and the basic patient data are shown in Table 1. The experiment was conducted in strict compliance with the Declaration of Helsinki, and all subjects signed an informed consent form.

### 2.3. Inclusion and Exclusion Criteria

Inclusion criteria are as follows: 3-7 d after the end of menstruation, with no sexual intercourse during this period; routine blood and white blood test results were normal; and age >22 years old.

Exclusion criteria are as follows: infertility caused by endocrine abnormalities in the woman and semen abnormalities in the men; the presence of acute inflammation of the internal and external genitalia and subacute or acute attacks of chronic inflammation; and vaginal bleeding.

### 2.4. Main Instruments and Reagents

Color Doppler ultrasound diagnostic instrument (GE Voluson E10, USA), transvaginal 4-dimensional ultrasound probe (GE RIC5-9-D, center frequency 5.0-9.0 MHz, USA), and Sonovir contrast agent (Bracco Suisse SA, SFDA Approval No. J20130045).

### 2.5. Testing Methods

Altogether 5 mL of saline was filled into the glass bottle with powdered Sonovir, and 2 mL was collected and added into 18 mL of saline to make 20 mL of Sonovir dilution solution. A routine 2D vaginal ultrasound was performed to clarify patients' bilateral ovaries, pelvis, and uterus (Figure 1); after routine disinfection and laying towels, a disposable silicone rubber double shot hysterosalpingogram tube was inserted vaginally into the uterine cavity, and 1.2-2.5 mL of saline was injected into the balloon. Subsequently, 5 mL of saline was extracted and injected into the subject's uterine cavity through the contrast tube to observe intrauterine polyps, myomas, and other occupancies or uterine adhesions. In 3D-HyCoSy, start the 3D mode prescan, keep the probe position fixed under the transverse uterine section, select the 3D mode after starting the contrast condition, adjust the pelvis to be echo-free, and adjust the sampling frame larger to ensure the observation range. The contrast dilution was injected slowly and uniformly into the uterine cavity, and the collection of 3D volume data was started when the two uterine horns became highly echogenic. After image acquisition, the pelvic and periovarian contrast distribution was observed via 2D contrast mode. The images are acquired 3 times continuously and stored for backup. When evaluation is needed, the images are pulled out, rotated, and cut, and the gain is adjusted for comprehensive analysis. For 4D-HyCoSy, in the center plane, start the contrast condition and 4D scan mode, turn down the gain, and turn up the sampling frame. During the process of contrast injection into the catheter, real-time dynamic observation of the high echo of contrast filling and flow in the uterine cavity and fallopian tubes is made to make a diagnosis, and the video can be played back frame by frame for analysis after being called up.

### 2.6. Results Assessment

All imaging results were reviewed by our two senior imaging physicians using a double-blind method, and subjects were analyzed for uterine, ovarian, and pelvic lesions and tubal patency based on 2D vaginal ultrasound, 3D-HyCoSy, and 4D-HyCoSy images. According to the Clinical Application Guideline of Ultrasonography in China, the subject's fallopian tubes were visualized throughout and traveled naturally, there was no resistance when pushing the contrast agent, the contrast agent was wrapped around the ovaries in a circular pattern, and the contrast agent was diffused evenly in the pelvis. Tubal development is discontinuous, local slender, nodular, or thickened, and there is resistance when injecting contrast medium, and after stopping injection of contrast medium, some contrast media recycle back to the inner orifice of the uterus (or even external orifice of the cervix). The contrast medium diffused slowly from the fallopian tube to the ovary and surrounded the ovary in an arc or semiring shape. The diffusion and sparse results of the contrast medium in the pelvic cavity were evaluated as tubal obstruction. The fallopian tube is not developed throughout the whole process (or only the proximal end of the fallopian tube), and the official cavity is slender, stiff, and curved. There was a great resistance when injecting the contrast medium. After stopping the contrast injection, almost all the contrast agent returned to the ectocervix and the external vaginal opening. It was evaluated as fallopian tube obstruction when there was no contrast agent around the ovaries and no contrast agent diffusion in the pelvis. When the results of the evaluation by two physicians were in dispute, the opinion of a third physician was sought.

### 2.7. Outcome Measures

The results of the FTRH examination [13] were employed as the gold standard to compare the effectiveness of different dimensions of the HyCoSy examination results in assessing the subjects for the presence of polyps, leiomyomas, and other occupancies in the uterine cavity or uterine adhesions. The calculation of diagnostic efficacy are as follows: both FTRH and this method were judged to be positive, regarded as true positive, and marked as*a*; both FTRH and this method were judged to be negative, regarded as true negative, and marked as*b*; FTRH is judged as positive, this method is judged as negative, it is regarded as false negative, and marked as*c*; FTRH is judged as negative, this method is judged as positive, it is regarded as false positive, and marked as*d*.Sensitivity = *a*/(*a* + *c*) × 100%; Specificity = *b*/(*b* + *d*) × 100%; Diagnostic accuracy = (*a* + *d*)/(*a* + *b* + *c* + *d*) × 100%.

### 2.8. Statistical Methods

Statistical analysis was performed using SPSS 22.0 software. The measurement data were recorded as ($\overset{-}{\chi }\pm s$), and the counting data were recorded as (%). Comparisons were made using the chi-square test, and differences were considered statistically remarkable at *P* < 0.05.

## 3. Results

### 3.1. Summary of Results

Vaginal ultrasound assessment of uterine cavity, pelvis, ovarian lesions, and tubal obstruction was moderately consistent with FTRH (Kappa = 0.616, 0.673, 0.654, and 0.640), 3D-HyCoSy was in good agreement with FTRH (Kappa = 0.812, 0.910, 0.906, and 0.894), and 4D-HyCoSy was in good agreement with FTRH (Kappa = 0.914, 0.903, 1.000, and 0.942), with 4D-HyCoSy being in good agreement with FTRH had the highest agreement.

### 3.2. Image Results

FTRH results manifested that uterine cavity lesions were detected in 18 patients, pelvic lesions in 11 cases, and ovarian lesions in 11 cases in 40 patients. A total of 80 fallopian tubes were found in 40 patients, and 71 tubal obstructions were examined by FTRH. Typical findings of vaginal ultrasound, 3D-HyCoSy, and 4D-HyCoSy are shown in Figures 2 and 3.

### 3.3. Comparison of Uterine Cavity Lesion Screening

Vaginal ultrasound detected 14 uterine cavity lesions with a diagnostic sensitivity of 50.00%, specificity of 77.27%, accuracy of 65.00%, and moderate concordance with FTRH (Kappa = 0.616, *P* < 0.05, Table 2). 3D-HyCoSy found 16 cases with a diagnostic sensitivity of 72.22%, specificity of 86.36%, accuracy of 80.00%, and good agreement with FTRH (Kappa = 0.812, *P* < 0.05, Table 3). 4D-HyCoSy discovered 17 cases with a diagnostic sensitivity of 94.44%, specificity of 100.0%, accuracy of 97.50%, and good agreement with FTRH (Kappa = 0.914, *P* < 0.05, Table 4).

### 3.4. Comparison of Pelvic Pathology Screening

16 pelvic lesions were tested by vaginal ultrasound, 10 pelvic lesions were found by 3D-HyCoSy, and 13 pelvic lesions were examined by 4D-HyCoSy. The diagnostic sensitivity, specificity, and accuracy of vaginal ultrasound were 63.64%, 64.52%, and 67.50%, respectively, with moderate agreement with FTRH (Kappa = 0.673, *P* < 0.05, Table 5). The diagnostic sensitivity, specificity, and accuracy of 3D-HyCoSy were 81.82%, 96.55%, and 92.50%, respectively, which were in good agreement with FTRH (Kappa = 0.910, *P* < 0.05, Table 6). The diagnostic sensitivity, specificity, and accuracy of 4D-HyCoSy were 90.91%, 89.66%, and 90.00%, respectively, which were in good agreement with FTRH (Kappa = 0.903, *P* < 0.05, Table 7).

### 3.5. Comparison of Ovarian Lesion Screening

9 ovarian lesions were tested by vaginal ultrasound, the diagnostic sensitivity was 45.45%, the specificity was 86.21%, and the accuracy was 75.00% (Kappa = 0.654, *P* < 0.05, Table 8). 12 ovarian lesions were found by 3D-HyCoSy, the diagnostic sensitivity was 90.91%, the specificity was 93.10%, and the accuracy was 92.50% (Kappa = 0.906, *P* < 0.05, Table 9). And 11 ovarian lesions were examined by 4D-HyCoSy, and it is completely consistent with the inspection results of FTRH (Kappa = 1, Table 10).

### 3.6. Comparison of Tubal Patency Test Results

Vaginal ultrasound detected 54 obstructions with a diagnostic sensitivity of 70.42%, specificity of 55.56%, accuracy of 68.75%, and moderate agreement with FTRH (Kappa = 0.640, *P* < 0.05, Table 11). 3D-HyCoSy found obstruction in 67 strips with a diagnostic sensitivity of 92.96%, specificity of 88.89%, accuracy of 92.50%, and good agreement with FTRH (Kappa = 0.894, *P* < 0.05, Table 12). 4D-HyCoSy identified obstruction in 68 entries with a diagnostic sensitivity of 95.77%, specificity of 100.0%, accuracy of 96.25%, and good agreement with FTRH (Kappa = 0.942, *P* < 0.05, Table 13).

## 4. Discussion

The fallopian tubes have the role of transporting sperm, picking up eggs, and being transported by fertilized eggs to the uterine cavity, and they occupy a dominant position among all the factors that cause infertility in women [14]. Thus, the correct and accurate assessment of tubal blockage is of great importance for the diagnosis and treatment of infertility. And for tubal obstruction assessment, both 3D-HyCoSy and 4D-HyCoSy also revealed superior results [15, 16]. However, few studies have been conducted to compare the effectiveness of 3D-HyCoSy with 4D-HyCoSy. Hence, this study is an essential reference for the further popularization of HyCoSy use. At the same time, for the increasing incidence of female infertility, finding the cause of infertility quickly and accurately is the key to complete clinical treatment and achieve normal pregnancy. By exploring the application of HyCoSy, it is also beneficial to better grasp the assessment of the causes of female infertility in the future, so as to provide patients with more reliable diagnosis and treatment advice.

In this study, we found that both 3D-HyCoSy and 4D-HyCoSy had better diagnostic results for infertility than 2D vaginal ultrasound, but the evaluation results of 4D-HyCoSy for uterine cavity, pelvis, ovarian lesions, and tubal patency were more consistent with laparoscopic tubal lavage, indicating that 4D-HyCoSy has a higher clinical application prospect. Previous studies have pointed out that although the clear images of 3D-HyCoSy provide a more visual and three-dimensional view of the course and morphology of the fallopian tubes, there are certain limitations, such as the fact that only one 3D image can be obtained per 3D-HyCoSy examination. And the start time and speed of the scan and the timing of the contrast agent need to be strictly controlled during the scan. At the same time, since the probe cannot be moved during 3D-HyCoSy, it is necessary to rely on the experience of the examiner to judge the depth, angle, and range of the scan, etc. Therefore, 3D-HyCoSy requires high professional skills of the operator, and only after proficiency can images of good quality be obtained [17–19]. The 4D-HyCoSy is a 3D volumetric database with high frame rate, which can display the whole process of contrast agent entering the uterine cavity from the catheter and developing the fallopian tubes in real time. The image is dynamic and clear, and it is convenient to observe the degree of patency of the fallopian tubes, the morphology of the tubal and uterine cavities, and the diffusion of contrast agent in the pelvis. The scanning process can rotate the plane to select the best viewing and acquisition angles [20, 21]. We believe that the reason for some discrepancies in the results of the two examinations may lie in the shorter image scanning time of 3D-HyCoSy, when a transient blockage and spasm of the fallopian tubes may have been caused by the accumulation of air bubbles, leading to misdiagnosis. Besides, 3D-HyCoSy is a posterior-to-forward sweep, and the position of the fallopian tubes needs to be predicted in relation to the uterus and ovaries to determine the time to activate the 3D mode; otherwise, the contrast agent may diffuse into the pelvis and interfere with the image or “off-target” the distal fallopian tubes [22]. Moreover, 3D-HyCoSy is susceptible to the influence of contrast agents that diffuse into the pelvis, parametrial venous reflux, and myometrium, and there are more confounding factors in the evaluation of the final results [23], while 4D-HyCoSy acquires a video recording that dynamically records the entire process of contrast medium entering the uterine cavity and flowing into the fallopian tube to its ejection from the umbilical end. Its advantage is that it allows dynamic observation and frame-by-frame playback, which is more conducive to clinical observation of the details of the fallopian tube and confirmation of the presence of diffusion and backflow [24]. Finally, the 4D-HyCoSy examination also allows the probe to be moved during the examination to find the most ideal viewing angle, thus allowing a more effective evaluation of the difference in bilateral fallopian tube visualization time [25]. Nevertheless, there are still several issues that deserve attention. For example, due to the lack of clinical guidelines for 4D-HyCoSy, some of the diagnostic criteria are still not quantified; there may be some subjective differences in the judgment of the results, which need to be evaluated in conjunction with patients' specific situation and physicians' opinion. In some children with severe tubal occlusion, the injected contrast agent may diffuse or return to other surrounding organs, so it should be pushed as slowly as possible to prevent reflux. If the uterus is positioned too far forward or backward, the position of the uterus can be adjusted by filling the bladder to prevent leakage of the contrast medium.

Of course, since this study is a retrospective analysis and the number of subjects is small, we cannot exclude that there may be chance in the test results. Subsequently, we need to conduct randomized controlled trials to further confirm the advantages and disadvantages of 3D-HyCoSy versus 4D-HyCoSy as soon as possible. In the meantime, we need to conduct a trial on the effect of infertility treatment under 4D-HyCoSy guidance to provide a more comprehensive reference for the future use of HyCoSy. Of course, the most critical point is that because neither 3D-HyCoSy nor 4D-HyCoSy has been widely used in clinical practice, there is a lack of unified clinical manipulation and evaluation guidelines for the evaluation of female infertility by 3D-HyCoSy and 4D-HyCoSy. This is also a big problem to realize the clinical application of 3D-HyCoSy and 4D-HyCoSy. Therefore, we hope that more researchers can join in the research on the diagnosis of female infertility by 3D-HyCoSy and 4D-HyCoSy and realize the popularization and use of 3D-HyCoSy and 4D-HyCoSy as soon as possible.

## 5. Conclusion

4D-HyCoSy can be used as an effective tool for clinical diagnosis of female tubal obstruction infertility and provide a reference basis for the design of subsequent clinical treatment plans.

## Figures and Tables

**Figure 1:** Saline hysterosalpingogram.

**Figure 2:** Female, 29 years old: (a) vaginal ultrasound reveals hydrosalpinx on the left fallopian tube. (b) 4D-HyCoSy examination reveals a contrast collection at the end of the left tubal dilatation.

**Figure 3:** Female, 32 years old: (a) endometrial polyp seen on vaginal ultrasound. (b) 3D-HyCoSy examination reveals endometrial polyps.

**Table 1:** Basic data of the subjects.

Patient information	*n*
Age	28.18 ± 3.66
Weight (kg)	55.58 ± 10.32
Height (cm)	158.65 ± 6.76
Family history of illness	
Have	2 (5.00)
None	38 (95.00)
History of miscarriage	
Have	4 (10.00)
None	36 (90.00)
Smoking	
Yes	8 (20.00)
No	32 (80.00)
Drinking	
Yes	7 (17.50)
No	33 (82.50)
Sleep situation	
Normal	16 (40.00)
Irregular	24 (60.00)
Place of residence	
City	29 (72.50)
Rural	11 (27.50)

**Table 2:** Diagnostic effectiveness of vaginal ultrasound and FTRH for uterine cavity lesions.

		FTRH		Total	Kappa	*P*
		(+)	(-)			
Vaginal ultrasound	(+)	9	5	14	0.616	<0.05
	(-)	9	17	26		
Total		18	22			

**Table 3:** Diagnostic effectiveness of 3D-HyCoSy and FTRH for uterine cavity lesions.

		FTRH		Total	Kappa	*P*
		(+)	(-)			
3D-HyCoSy	(+)	13	3	16	0.812	<0.05
	(-)	5	19	24		
Total		18	22			

**Table 4:** Diagnostic effectiveness of 4D-HyCoSy and FTRH for uterine cavity lesions.

		FTRH		Total	Kappa	*P*
		(+)	(-)			
4D-HyCoSy	(+)	17	0	17	0.914	<0.05
	(-)	1	22	23		
Total		18	22			

**Table 5:** Diagnostic effectiveness of vaginal ultrasound versus FTRH for pelvic lesions.

		FTRH		Total	Kappa	*P*
		(+)	(-)			
Vaginal ultrasound	(+)	7	9	16	0.673	<0.05
	(-)	4	20	24		
Total		11	29			

**Table 6:** Diagnostic effectiveness of 3D-HyCoSy versus FTRH for pelvic lesions.

		FTRH		Total	Kappa	*P*
		(+)	(-)			
3D-HyCoSy	(+)	9	1	10	0.910	<0.05
	(-)	2	28	27		
Total		11	29			

**Table 7:** Diagnostic effectiveness of 4D-HyCoSy versus FTRH for pelvic lesions.

		FTRH		Total	Kappa	*P*
		(+)	(-)			
4D-HyCoSy	(+)	10	3	13	0.903	<0.05
	(-)	1	26	27		
Total		11	29			

**Table 8:** Diagnostic effectiveness of vaginal ultrasound and FTRH on ovarian lesions.

		FTRH		Total	Kappa	*P*
		(+)	(-)			
Vaginal ultrasound	(+)	5	4	9	0.654	<0.05
	(-)	6	25	31		
Total		11	29			

**Table 9:** Diagnostic effectiveness of 3D-HyCoSy and FTRH on ovarian lesions.

		FTRH		Total	Kappa	*P*
		(+)	(-)			
3D-HyCoSy	(+)	10	2	12	0.906	<0.05
	(-)	1	27	28		
Total		11	29			

**Table 10:** Diagnostic effectiveness of 4D-HyCoSy and FTRH on ovarian lesions.

		FTRH		Total	Kappa	*P*
		(+)	(-)			
4D-HyCoSy	(+)	11	0	11	1.000	<0.05
	(-)	0	29	29		
Total		11	29			

**Table 11:** Diagnostic effectiveness of vaginal ultrasound versus FTRH for tubal obstruction.

		FTRH		Total	Kappa	*P*
		(+)	(-)			
Vaginal ultrasound	(+)	50	4	54	0.640	<0.05
	(-)	21	5	26		
Total		71	9			

**Table 12:** Diagnostic effectiveness of 3D-HyCoSy versus FTRH for tubal obstruction.

		FTRH		Total	Kappa	*P*
		(+)	(-)			
3D-HyCoSy	(+)	66	1	67	0.894	<0.05
	(-)	5	8	13		
Total		71	9			

**Table 13:** Diagnostic effectiveness of 4D-HyCoSy versus FTRH for tubal obstruction.

		FTRH		Total	Kappa	*P*
		(+)	(-)			
4D-HyCoSy	(+)	68	0	68	0.942	<0.05
	(-)	3	9	12		
Total		71	9			

## Data Availability

The datasets used and analyzed in the current study would be available from the corresponding author upon request.

## References

[1] Carson S. A., Kallen A. N. (2021). Diagnosis and management of infertility: a review. *Journal of the American Medical Association*.

[2] Vander Borght M., Wyns C. (2018). Fertility and infertility: definition and epidemiology. *Clinical Biochemistry*.

[3] Starc A., Trampus M., Pavan Jukic D., Rotim C., Jukic T., Polona M. A. (2019). Infertility and sexual dysfunctions: a systematic literature review. *Acta Clinica Croatica*.

[4] Infertility Workup for the Women’s Health Specialist (2019). Infertility workup for the women’s health specialist. *Obstetrics and Gynecology*.

[5] Neven A. C. H., Laven J., Teede H. J., Boyle J. A. (2018). A summary on polycystic ovary syndrome: diagnostic criteria, prevalence, clinical manifestations, and management according to the latest international guidelines. *Seminars in Reproductive Medicine*.

[6] Bala R., Singh V., Rajender S., Singh K. (2021). Environment, lifestyle, and female infertility. *Reproductive Sciences*.

[7] Dishuck C. F., Perchik J. D., Porter K. K., Gunn D. D. (2019). Advanced imaging in female infertility. *Current Urology Reports*.

[8] Li Q. Y., Zhou X. L., Qin H. P., Liu R. (2004). Analysis of 1006 cases with selective salpingography and fallopian tube recanalization. *Zhonghua Fu Chan Ke Za Zhi*.

[9] Miyazaki T., Kobayashi T., Kuji N. (1995). Evaluation of the radiologic findings on hysterosalpingography by selective hydrotubation with flexible hysterofiberscope. *Journal of Assisted Reproduction and Genetics*.

[10] Boned-Lopez J., Alcazar J. L., Errasti T. (2021). Severe pain during hysterosalpingo-contrast sonography (HyCoSy): a systematic review and meta-analysis. *Archives of Gynecology and Obstetrics*.

[11] Hong Q., Cai R., Chen Q. (2017). Three-dimensional HyCoSy with perfluoropropane-albumin microspheres as contrast agents and normal saline injections into the pelvic cavity for morphological assessment of the fallopian tube in infertile women. *Journal of Ultrasound in Medicine*.

[12] Gu P., Yang X., Zhao X., Xu D. (2021). The value of transvaginal 4-dimensional hysterosalpingo-contrast sonography in predicting the necessity of assisted reproductive technology for women with tubal factor infertility. *Quantitative Imaging in Medicine and Surgery*.

[13] Yapca O. E., Delibas I. B., Karaca I., Kumtepe Y., Kadanali S. (2015). Time-limited hydrotubation combined with clomiphene citrate treatment for unexplained infertility. *Clinical and Experimental Obstetrics & Gynecology*.

[14] Bosdou J. K., Konstantinidou E., Anagnostis P., Kolibianakis E. M., Goulis D. G. (2019). Vitamin D and obesity: two interacting players in the field of infertility. *Nutrients*.

[15] Robertshaw I. M., Sroga J. M., Batcheller A. E. (2016). Hysterosalpingo-contrast sonography with a saline-air device is equivalent to hysterosalpingography only in the presence of tubal patency. *Journal of Ultrasound in Medicine*.

[16] Luong E., Ludwin A., Winter T. (2020). Saline-air hysterosalpingo-contrast sonography is equivalent to the modified hysterosalpingogram following hysteroscopic sterilization. *Ultrasound Quarterly*.

[17] Wang J., Li J., Yu L., Han S., Shen X., Jia X. (2017). Application of 3D-HyCoSy in the diagnosis of oviduct obstruction. *Experimental and Therapeutic Medicine*.

[18] Gao Y. B., Yan J. H., Yang Y. D., Sun J., Dong J. Y., Cui G. H. (2019). Diagnostic value of transvaginal four-dimensional hysterosalpingo-contrast sonography combined with recanalization in patients with tubal infertility. *Nigerian Journal of Clinical Practice*.

[19] Liang N., Wu Q. Q., Li J. H., Gao F. Y., Sun F. L., Guo C. X. (2019). Causes of misdiagnosis in assessing tubal patency by transvaginal real-time three-dimensional hysterosalpingo-contrast sonography. *Revista da Associação Médica Brasileira*.

[20] Bisogni F. A., Galanti F., Riccio S. (2021). 4D-HyCoSy performed in a reproductive center: retrospective analysis of pain perception, complications and spontaneous pregnancy rate after the technique. *European Review for Medical and Pharmacological Sciences*.

[21] Liu Y., Zhang N., He Y. (2020). Spontaneous conception outcome in infertile women after four-dimensional hysterosalpingo-contrast-sonography. *BMC Pregnancy Childbirth*.

[22] Chan C. C., Ng E. H., Tang O. S., Chan K. K., Ho P. C. (2005). Comparison of three-dimensional hysterosalpingo-contrast-sonography and diagnostic laparoscopy with chromopertubation in the assessment of tubal patency for the investigation of subfertility. *Acta Obstetricia et Gynecologica Scandinavica*.

[23] Watermann D., Denschlag D., Hanjalic-Beck A., Keck C., Karck U., Prompeler H. (2004). Hystero-Salpingo-Kontrastsonographie mit 3D-Ultraschall: eine Pilotstudie. *Ultraschall in der Medizin-European Journal of Ultrasound*.

[24] Chen L. S., Zhu Z. Q., Li J. (2020). Hysterosalpingo-contrast-sonography vs. magnetic resonance- hysterosalpingography for diagnosing fallopian tubal patency: a systematic review and meta-analysis. *European Journal of Radiology*.

[25] Chen S., Du X., Chen Q., Chen S. (2019). Combined real-time three-dimensional hysterosalpingo-contrast sonography with B mode hysterosalpingo-contrast sonography in the evaluation of fallopian tube patency in patients undergoing infertility investigations. *BioMed Research International*.

